The article "Identification for surrogate drought tolerance in maize inbred lines utilizing high-throughput phenomics approach" was retracted in 2022. Reasons: compromised peer review; a conflict of interest; concerns about the authorship.

# Identification for surrogate drought tolerance in maize inbred lines utilizing high-throughput phenomics approach

**DOI:** 10.1371/journal.pone.0254318

**Published:** 2021-07-27

**Authors:** Zahoor A. Dar, Showket A. Dar, Jameel A. Khan, Ajaz A. Lone, Sapna Langyan, B. A. Lone, R. H. Kanth, Asif Iqbal, Jagdish Rane, Shabir H. Wani, Saleh Alfarraj, Sulaiman Ali Alharbi, Marian Brestic, Mohammad Javed Ansari

**Affiliations:** 1 Dryland Agricultural Research Station, Sher-e-Kashmir University of Agricultural Sciences &Technology-Kashmir, Rangreth Srinagar, Jammu and Kashmir, India; 2 Department of Entomology, Sher-e-Kashmir University of Agricultural Sciences & Technology of Kashmir, Srinagar-Kargil, Ladakh, India; 3 Department of Biotechnology, University of Agricultural Sciences, Bangalore, India; 4 ICAR-National Bureau for Plant Genetic Resources, New Delhi, India; 5 Department of Agronomy, Sher-e-Kashmir University of Agricultural Sciences &Technology-Kashmir, Srinagar, Jammu and Kashmir, India; 6 Department of Agronomy, Sher-e-Kashmir University of Agricultural Sciences &Technology-Kashmir, Wadura Sopore, Jammu and Kashmir, India; 7 Department of Soil Science, Sher-e-Kashmir University of Agricultural Sciences &Technology-Kashmir, Srinagar, Jammu and Kashmir, India; 8 Department of Drought Science, ICAR-NIASM, Baramati, New Delhi, India; 9 MRCFCF, Sher-e-Kashmir University of Agricultural Sciences &Technology-Kashmir, Srinagar, Jammu and Kashmir, India; 10 Zoology Department, College of Science, King Saud University, Riyadh, Saudi Arabia; 11 Department of Botany & Microbiology, College of Science, King Saud University, Riyadh, Saudi Arabia; 12 Department of Plant Physiology, Slovak University of Agriculture, Nitra, Slovakia; 13 Department of Botany, Hindu College Moradabad (Mahatma Jyotiba Phule Rohilkhand University Bareilly), Moradabad, India; Ghazi University, PAKISTAN

## Abstract

Screening for drought tolerance requires precise techniques like phonemics, which is an emerging science aimed at non-destructive methods allowing large-scale screening of genotypes. Large-scale screening complements genomic efforts to identify genes relevant for crop improvement. Thirty maize inbred lines from various sources (exotic and indigenous) maintained at Dryland Agriculture Research Station were used in the current study. In the automated plant transport and imaging systems (LemnaTec Scanalyzer system for large plants), top and side view images were taken of the VIS (visible) and NIR (near infrared) range of the light spectrum to capture phenes. All images were obtained with a thermal imager. All sensors were used to collect images one day after shifting the pots from the greenhouse for 11 days. Image processing was done using pre-processing, segmentation and flowered by features’ extraction. Different surrogate traits such as pixel area, plant aspect ratio, convex hull ratio and calliper length were estimated. A strong association was found between canopy temperature and above ground biomass under stress conditions. Promising lines in different surrogates will be utilized in breeding programmes to develop mapping populations for traits of interest related to drought resilience, in terms of improved tissue water status and mapping of genes/QTLs for drought traits.

## Introduction

Modern agriculture is facing challenges of producing sufficient food [1–3] for a global population expected to reach 9.7 billion by 2050 [4, 5]. In the past several decades, the major food crop production has increased considerably as a result of timely application of fertilizers and other inputs, improved farming practices [6, 7] and genetic improvement [8].

Despite increased food production, mounting human population leads to a continued gap between demand and supply of food grains [9]. Plant phenomics can play a major role in lessening this gap by providing large scale and high throughput phenotyping facilities for crop breeding.

Yang et al. [10] reported that advanced plant phenomics would facilitate efficient use of genetic data and eventually direct to novel gene discovery and enhanced crop yield and quality in the field. Furthermore, the acquisition of comprehensive phenotypic data has become one of the major bottlenecks impeding crop breeding and functional genomics studies. However, the recent technological support to bypass many hindrances to direct the extensive advanced methods for broad-scale phenotyping had led to data achievements and processing in the 21^st^ century.

Plant phenomics starts with; i) identification of a desired trait such as a specific stress or any particular physiological process, ii) data estimation from devices, i.e., imaging devices and iii) calculation of the results to give response to the extracted data. The first step is done with the help of high throughput phenotyping platforms or phenomic tools. The second and third steps depend on computing methods [11]. High-throughput plant phenotyping examines temporal plant image sequences taken by multimodal cameras at regular intervals under a range of stresses, e.g., drought, salinity and heat stress. The high-performance phenotyping is widespread and supports automated analysis of large data samples associated with the development of image registration systems in various spectral regions. In advanced techniques, it approaches to cultivating plant objects under standardized conditions, employing sensory technologies, robotics and methods for data processing and analysis through computer vision and machine learning (artificial neural network) [12]. The image sequences captured can help in computing structural or morphological identification of plant phenotypes. They are further categorised into holistic and component phenotypes. The holistic phenotypes are used to work out its basic geometrical characteristics [13, 14]. The component phenotypes are figured out by examining individual components of the plants such as length of leaf, leaf chlorophyll content, stem angle, size of flower and fruit volume [14–18]. Traditional phenotyping methods dealing with plant characteristics couldn’t aid in systematic functional analysis and have resulted into functional map between genotype and phenotype [19]. This is often because of adequate data available on plant phenotype to foresee such relations with greater power. Spotlight on overcoming these pitfalls has led to a promising and incomparable transdisciplinary area of research termed “phenomics” [20].

Phenomics tools facilitate high-throughput phenotyping for crop improvement to cope with present and future demographic and climate change scenarios. Phenomics has evolved as a novel area of biology that involves high-dimensional phenotypic data at multiple steps of organization for full characterization of the complete set of phenotypes of a genome. High-throughput phenotyping is a new frontier designed for crop improvement involving association of various approaches to determine the plant phenotype to genetic expression for elucidating the concerns regarding future food and nutritional security under declining natural resources and climate unpredictability. This non-destructive process refers to sensing and quantifying same plant traits repeatedly and helps in phenotype computation by analysing captured images of a large number of plants with precision in a short time interval [14].

High-throughput phenotyping technologies are being effectively used due to; a) automated, non-destructive method with online assessment of multiple morpho-physiological plant traits; b) time-series measurements essential for following the growth sequence, plant performance and plant stress response at high-resolution and c) reduced cost, labour, and time for analyses with automation, remote sensing, improved data integration and experimental design [21–23]. Destructive phenotyping methods including harvesting plant responses for assessment of water relations and other physiological responses to stresses limit our studies to very few plants and make this exercise cost and labour intensive. Several equipment, for instance, photosynthetic meters, stomatal conductance meter, SPAD meter, chlorophyll fluorescence meter, NDVI sensors have evolved as versatile tools for physiologists, plant breeders and agronomists for conducting field investigations. The existing phenotyping platforms comprise of a number of imaging techniques to achieve high-throughput non-destructive data on plant phenotype for quantitative studies of complex traits [24]. Here, an effort has been made to highlight non-invasive methods utilizing images for analysing plant responses to drought stress. These methods are based on images captured by background system that senses different bands of wavelength in electromagnetic spectrum. They include visible, infrared, fluorescence, NIR/SWIR and hyper-spectral/multispectral imaging techniques.

Maize plants adjust leaf positioning (i.e., phyllotaxy) in reaction to light signals perceived through the photochrome pathway in order to optimize light interception [25]. Automated phenotyping analysis has made it possible to investigate how diverse maize inbred lines changed their phyllotaxy at different developmental stages.

New derived holistic phenotype, namely, bi-angular convex-hull area ratio (*BA_CH_R*), is defined as:

$$BA_{CH}R=\frac{AreaCH_{at\;side\;view\;0{}^{\circ}}}{AreaCH_{at\;side\;view\;90{}^{\circ}}}$$

Whereas, *Area*_*CH*_ is the area of the convex-hull.

Variation in canopy architecture influences the proportion of incident solar radiation, which can be intercepted by leaves; thus, influences the proportion of the energy which can be converted to chemical energy [10]. Increases in field planting density over the last century have shifted the ideal ideotype of maize plants towards more erect leaf angles. Leaf erectness has been traditionally assessed by calculating the angle between a specifically defined leaf and the plant stem [12]. High planting densities also activate the response to shade avoidance, causing plants to spend more energy in stem elongation at the cost of yield [14]. Artificial selection for yield at high planting densities has also driven a reduction in the shade avoidance response of maize hybrids, likely also mediated through the phytochrome path-way, an alternative derived holistic phenotype called as plant aspect ratio (*PAR*) that combine data on plant height and leaf extent. *PAR* is defined as:

$$PAR=\frac{Height\;BR_{at\;side\;view}}{Diameter\;MEC\;at\;top\;view}$$

Whereas, height _*BR*_ and diameter _*MEC*_ denote the height of the bounding rectangle (BR) of the plant in side view 0^0^, and the diameter of the minimum enclosing circle (MEC) of the plant in top view, respectively [26]. The objective of the present study was to use above two ratios along with other image-based surrogates to derive the results on the variability in tissue water status among maize inbred lines. Furthermore, using high-throughput phenotyping in association with environmental and field conditions would be used for post-harvest yield and quality assessment in the future.

## Materials and methods

### Plant material

Thirty maize inbred lines (Appendices 1 & 2) from different sources (exotic and indigenous) maintained at Dryland Agriculture Research Station (SKUAST- Kashmir) were chosen for the study.

**Appendix 1:** List of maize inbred lines used in the study.

**S. No**	**Line**	**Source**
1.	CML-425	CIMMYT, Mexico
2.	CML-474	
3.	CML-470	
4.	CML-286	
5.	KDM-926B	DARS, Budgam
6.	KDM-895A	
7.	KDM-914A	
8.	KDM-340A	
9.	KDM-362A	
10.	KDM-916A	
11.	KDM-930A	
12.	KDM-954A	
13.	KDM-944A	
14.	KDM-963A	
15.	KDM-921A	
16.	KDM-892A	
17.	KDM-932A	
18.	KDM-332A	
19.	KDM-927A	
20.	KDM-343A	
21.	V-351	VPKAS, Almora
22.	V-335	
23.	NGB-17097-1	Nordic Gene Bank, Sweden
24.	NGB-17097	
25.	NGB-17094-1	
26.	NGB-17096-1	
27.	NGB-17095-1	
28.	NGB-17099-1	
29.	KDM-1095	DARS, Budgam
30.	KDM-1156	

**Appendix 2:** Genotype names corresponding to the genotype IDs used in the dataset.

**Gen ID**	**Inbred**	**Gen ID**	**Inbred**
1	CML-425	16	KDM-892A
2	CML-474	17	KDM-932A
3	CML-470	18	KDM-332A
4	CML-286	19	KDM-927A
5	KDM-926B	20	KDM-343A
6	KDM-895A	21	V-351
7	KDM-914A	22	V-335
8	KDM-340A	23	NGB-17097-1
9	KDM-362A	24	NGB-17097
10	KDM-916A	25	NGB-17094-1
11	KDM-930A	26	NGB-17096-1
12	KDM-954A	27	NGB-17095-1
13	KDM-944A	28	NGB-17099-1
14	KDM-963A	29	KDM-1095
15	KDM-921A	30	KDM-1156

### Growth conditions

Plants were grown in 12-cm diameter plastic pots (Nisarga 302) filled with 8 kg of clay-loam soil under natural conditions with average temperature of 30°C. Four healthy seeds were sown in each pot and later reduced to one seedling in each pot. After 30 days of sowing, pots were shifted to greenhouse maintained at 32/24°C day/night temperature, 50–65% relative humidity and 450–750μmol m^-2^s^-1^ PAR. Two pots were maintained for well-watered and water stressed treatments for each genotype throughout the experiment.

### Assessment of soil field capacity

The soil was air-dried and ground to pass through a 5 mm sieve at room temperature for determining field capacity (FC). Water holding capacity was assessed using a gravimetric method [27]. Five pots were randomly selected and kept in tray containing water and the soil was allowed to absorb water through drainage holes at the bottom of the pots by capillary action overnight. The wet surface on the top layer of the soil was considered as an indicator of completion of capillary action and hence absorption of soil moisture up to the FC. Then excess water was allowed to drain by moving the pots carefully to empty trays without water until there was no sign of water dripping from the pots. The FC was calculated based on initial dry and final weights of the pots. The pots were weighed every day and the reduction in pot weight was used to calculate relative water losses. Nearly 70% and 40% of water at FC were maintained in well-watered and water-stressed treatments, respectively.

### Measurement of shoot fresh and dry weights

Fresh weight (g) of plants was determined on single-plant basis after 45 days of sowing with above ground parts. After the plant parts get dried and attained constant weight, dry weight was measured.

### Controlled phonemics facility

#### Watering and weighing of plants

In the automated plant phenotyping platforms, plants were watered at watering/weighing station using peristaltic pumps that supply water or nutrient solutions either as a pre-defined fixed volume or as an individually calculated amount as the difference of a carrier (including pot) weight to a pre-defined target weight. In order to optimize the watering regime for maize growth, top watering was preferred over bottom watering for retaining moisture in the soil. Water used by plants per day was determined as a difference between the pot weight after watering on previous day and the same before watering on a particular day. There was no mineral deposition and growth of algae on the soil surface that could affect the quality of image background seen as particle fluorescent signals. During watering (target volume) with the HT system, both weights before and after watering were measured and recorded in the database to estimate water consumption by plants per day. These values were used for estimating ratio of biomass produced at the end of the experiment and water consumed per day (RBMU).

#### Image acquisition

At ICAR-NIASM, the high-throughput (HT) automated non-invasive phenotyping (LemnaTec) system having a capacity to phenotype midsized to large plants using three imaging sensors, i.e., infrared (IR), visible (VIS) and near infrared (NIR) imaging were used to capture phenotypic variation in the plants. Weighing and watering is carried out in an automatic approach (Fig 1).

**Fig 1:** LemnaTec plant phenomics facility at NIASM, Baramati.

In the automated conveyer for plant transport and imaging systems (ICAR-NIASM Lemna Tec Scanalyzer system for large plants), top and side view images were acquired in VIS and NIR light spectrum (Fig 1). These images were captured using piA2400-17gc CCD cameras (Basler, Ahrens-burg, Germany) with top and side illumination of plants through incandescent bulbs (FQ24W865HO or FH28W865HE, respectively, OsramGmbH, München Germany). Images captured from 9^th^ January to 19^th^ January 2018 (Day 02-Day 11) were analysed. Images were collected once per day for 11 days. Imaging started one day after shifting the pots from the greenhouse. The dataset is planned to aid in generating new computer vision algorithms in order to extract holistic phenotypic parameters explicitly from maize and to facilitate identification of surrogates for differentiating control and stress treatments. The folder for each plant is named as Plant ID-genotype ID. Appendix 1 and show genotype names corresponding to the genotype IDs used in the dataset. Each folder is subdivided into three subfolders, namely, side view 0^0^, side view 90^0^ and top view.

#### Image processing

The Lemnagrid, integrated analysis software for high-throughput plant image analyses was used for image-based plant feature extraction. Image processing was done in two sequential steps, i.e., image segmentation and feature extraction. A colour image from a VIS camera was transformed from RGB to LAB colour space for separate out foreground from the background. Threshold was applied individually on both grey scale images from the output channels *A* and *B*. The result were two binary images, which were combined and refined using logical set operation (OR) and general morphological operations (erosion, dilation, fill). The final image mask was used to measure the size of the projected area of a plant by counting the number of image pixels. These pixels were being used to estimate the volume by using following formula:

Volume=topviewarea×sideviewarea(1)×sideviewarea(2)

#### Canopy temperature measurement and analysis

Canopy temperature was calculated between 10:00 and 14:00 h on sunny, cloudless days on all genotypes from the centre of each plot’s canopy surface. In order to reduce the confounding effects of environmental variations on genotypic performance over this 4 h period, CT measurements were taken from one replication of all genotypes in about 20 min. All thermal images were taken by thermal imager (Vario CAM hr Inspect 575, Jenoptic, Germany) that works in the wavebands of 8–14 μm, having a thermal resolution of 0.01°C and capacity to produce images with spatial resolution of 768 × 576 pixels. A hand operated track mounted trolley was used for imaging purpose. Thermal camera was used to make sure that constant distance (about 1m) and angle between the camera and canopy should be maintained while taking all the measurements. Dry and wet references were used to mimic leaves with fully closed and fully open stomata, respectively [28] and to circumvent extreme conditions while image is captured. Measurements consisted of one image per plot three to four times from R1 through R6 stage. The IR image was captured at 3–5-day interval. For analysis of captured images and their storage, IRBIS® software (Jenoptic, Germany) was used. Emissivity for measurements of leaves and plant canopies was set at 0.96. The areas of interest for analysis in the imager’s software were outlined to obtain the minimum CT of the entire field of view of the infrared camera. Mean of average temperature for the period of 10.00 to 14.00 hr of the day was considered as mean environment temperature. Canopy temperature depression (CTD) was worked out by subtracting mean environment temperature from the canopy temperature.

## Results

For identification of drought tolerance, we used high-throughput phenomics (HTP) approach to determine various favarouble aspects which may enhance the yield besides disfavour the drought stress in maize inbred lines. Based on different image-based features, the analysed results for the plant aspect ratio in control and stress plots, bi angular convex-Hull area ratio in control and stress plots were deterimned (Figs 2A, 2B, 3A, 3B). The median value of bi-angular convex-hull area rato for all inbred lines was in the range of 1.40 to 4.83 in control and 1.06 to 4.23 in stressed plants. The lines showing the highest values for the ratio in control and stressed pots were KDM-1156 and KDM-926B, respectively.

**Fig 2:** Aspect ratio in control (a) and water stressed pots (b).

**Fig 3:** Bi-angular convex-hull area ratio in control (a) and water stressed pots (b).

Fig 4A–4D shows the average plant aspect ratio for all plants of each of 30 inbred lines through day 2 to day 11. It is evident from the figure that the plant aspect ratio for the inbred lines shows steep decrease in control as compared to several ups and downs in stressed pots with time, since the rate of increase in plant width is more compared to the plant height.

**Fig 4:** Illustration of genetic regulation of plant aspect ratio in control (a) and stressed pots (b), and genetic regulation of bi-convex hull ratio in control (c) and stressed pots (d).

Plant aspect ratio is a derived trait calculated from the combination of plant height and diameter and it is the ratio between the maximum length to maximum width. Plant aspect ratio identifies potential differences in the canopy architecture, which would be produced by different crop accessions in the field. The median value of plant aspect ratio for all inbred lines was within 0.75–1.33 and 0.41–0.95 in control and stressed pots. Lines showing maximum values for the ratio in control and stress pots were V-351 and KDM-926B (Figs 5 and 6).

**Fig 5:** Top ranking aspect ratio lines in control and stressed pots.

**Fig 6:** Top ranking bi-convex hull ratio lines in control and stressed pots.

The estimated heritability-the proportion of total variation elucidated by genetic variation for bi-angular convex-hull area ratio was moderate, signifying that the observed rotation is partially under the direct control of genes and is likely to be also regulated by environmental factors as well as genotype by environment interactions. The micro-environment variance as non-heritable portion is attributed to inaccuracy by software; however, the plant architecture phenotyping at more mature stages of development is more precise and highly predictive compared to early developmental stage.

Amongst the other surrogates predicted from the study besides the above mentioned include area, boundary point count, boundary point roundedness, calliper length and centre of mass to boundary distribution, compactness, convex hull circumference, mean colour red and object sum Area. These surrogates differentiated the inbred lines between control and stress conditions except KDM-340A in area, CML-286, CML-470 in boundary point count, boundary point roundedness, calliper length, centre of mass to boundary distribution and compactness, and V-351 for convex hull circumference, mean colour red, object sum area and minimum enclosing circle diameter. The relationship between different surrogates and biomass in control and stressed pots shows stronger association in all surrogates in control as compared to stressed plants except area, which has association significant in both situations (Figs 6 & 7). Two new holistic phenes were observed in the study, i.e., bi-angular convex-hull area ratio and plant aspect ratio. Bi-angular convex-hull area ratio is defined as the ratio of the convex-hull area of the plant when observed from the side at a particular angle and the convex-hull of the same plant when looked at a rotation of 90° angle. Variations in bi-angular convex-hull area ratio provide information regarding temporal change in phyllotaxy.

**Fig 7:** Relationship between surrogates and biomass in control (a) and stressed plants (b).

We observed that a strong association was found between canopy temperature and above ground biomass under stress conditions. Results revealed that inbred lines with lower canopy temperature had relatively higher yield under stress regime (Figs 8 & 9). Though, under normal irrigated conditions, constant correlation between canopy temperature and biomass was not observed. Overall, the inferences drawn from studies cleared those genotypes that maintain cooler canopies produce higher yield.

**Fig 8:** Relationship between canopy temperature and biomass in control plants.

**Fig 9:** Relationship between canopy temperature and biomass in stressed plants.

## Discussion

Maize is the most important and major crop to support life, but the yield is strongly threatened by drought stress [29]. The drought tolerance has been introduced by plant breeders using many approaches, including molecular breeding systems [30], transgenes, marker assisted selection, genome editing and multi-parent advanced generation intercross [31]. All these approaches have focussed to enhance the yield and increase the drought stress in maize until harvesting. For identification of drought tolerance in maize, high-throughput phenomics (HTP) approach was used to determine various favarouble aspects which may enhance the yield. Based on different image-based features a significant differences were found in bi angular convex-Hull area ratio. The microenvironment variation act as a non-heritable portion of variance comprises of some percent of inaccuracy in quantification created by the software itself [12]. This micro-variation suggests that full-grown maize plant architecture require phenotyping at more mature stages of development. Since the early developmental stage, measurements have only moderate predictive value at later stages in development [29]. The inbred lines, which showed maximum values for the aspect ratio were KDM-1156 and KDM-926B. Plant aspect ratio is a trait determined from plant height and diameter. Plant aspect ratio identifies the potential differences in the canopy architecture. It is also to be noted that some inbred lines have higher plant aspect ratios than others. These inferences noticeably showed the potential of plant aspect ratio to be an effective phenotype regulated by genetic variation [4]. The canopy temperature is an exceptional marker for crop water status estimation and act as a selection criterion for spotting of genotypes tolerant to water deficit conditions [32]. Infrared Thermal Imaging technique estimated the genotypic variation among maize inbred lines, therefore enhancing the breeding programs for drought tolerance of maize under temperate conditions of Kashmir, a way forward. The modules like thermal infrared thermometers and remote thermal imaging systems are useful in determining canopy temperatures in plant phenotyping [12]. However, in present study the canopy temperature successfully indicated the values of biconvex hull ratio, aspect ratios, water use efficiency, and response of different surrogates to drought stresses. Further, the genotypes that maintain cooler canopies during water stress may produce higher yield; showing that the cooler canopies help in producing higher yields [33] under drought stress.

## Conclusion

In conclusion, the findings provide a basis and future directions of research for planning a robust breeding programme to develop maize inbred lines tolerant towards drought stress involving mapping maize populations harbouring various traits of interest related to drought resilience. Issues in field phenotyping potential limit our propensity to dissect the genetics of quantitative traits, especially those concerned to drought tolerance. Enhancing crop yield under water-limited environments is most intimidating challenge faced by breeders. The effective field-based high-throughput phenotyping platforms (HTPPs) remain a bottleneck for future breeding advances. The recent advances in field HTPPs at an affordable cost, high capacity for data recording, scoring and processing, and non-invasive remote sensing methods, together with automated environmental data collection help in evaluating the yield and other quality parameters in maize under drought stress. The analysis of key plant parts and features may complement direct phenotyping under field conditions and the improvements in user-friendly data management strategy with a more powerful interpretation of results, which had increased the use of field HTPPs in bumper production of maize in drought prone areas. Therefore, increasing the efficiency of crop genetic improvement to meet the needs of foods for future generations are based on the principles and broad set of references useful for the management of phenotyping practices. Therefore, the study and genetic dissection of drought tolerance in maize will help in development and release of drought-tolerant cultivars.
